# On Gesell Evaluation System for Disabled Children in Minority Areas

**DOI:** 10.1155/2022/4210116

**Published:** 2022-01-25

**Authors:** Guozhi Chen, Weiwei Tan, Yu Shi, Ming Chen, Qin Huang, Yingying Lin, Jinsheng Jiang, Wen-Lung Chang, Yanzhi Huang

**Affiliations:** ^1^Guangxi Zhuangzhu Autonomous Region Disabled Rehabilitation Research Center, Nanning, China; ^2^School of Education Science, Nanning Normal University, Nanning, China

## Abstract

This paper takes 105 disabled children from the Disabled Rehabilitation Research Center of the South China minority autonomous region as the survey objects. Based on the Gesell scale, it collects health data such as exercise ability and health status of disabled children, analyzes the data in accordance with SPSS software, and constructs comprehensive disease analysis model of 105 disabled children. Moreover, according to five indicator data collected and tested for disabled children (adaptability, big movements, fine movements, language, and personal-social) in Gesell scale, comprehensive disease indicators of the disabled children are calculated and statistically analyzed together with age and gender information. This study analyzed comprehensive diseases and the correlation among various indicators, concluding that most disabled children aged 3–7 are diagnosed with moderate and severe developmental retardation, and retardation level is in obvious normal distribution. At the same time, there is a significant correlation between indicators of ability test interval and measurement indicators with age. This study suggests that targeted treatment and rehabilitation plans should be implemented for disabled children of different ages according to different indicators of ability test interval, which has reference value and significance for improving the treatment level of disabled children and realizing targeted rehabilitation.

## 1. Introduction

Limited by regional economy, health and culture, and other factors, minority areas have always lagged behind other areas. It is difficult for them to effectively utilize existing child health resources, especially ethnic minorities in remote border areas, so health level of children is far below the national average [1].

To be specific, in South China, according to the 2019 census data, developmental health problems of children in minority areas were severe, and disability-related incidence rate reached 5.6%, which was more than double the overall average (2.1%). Obviously, disability has severely affected overall population quality and economic and social development there. Therefore, an important issue in enhancing living standards of minority areas is about how to provide better treatment and rehabilitation for disabled children in these areas [2, 3].

In order to improve the level of treatment and rehabilitation, this study believes a key step is to deeply and systematically understand relevant factors that affect healthy development of disabled children. As an essential tool for evaluating and measuring development of children, Gesell scale can identify neuromuscular or sensory systems are defective or not and find developmental abnormalities that can be treated, as well as subsequent changes in behaviors of high-risk children.

In summary, it is useful for diagnosing autism and developmental retardation. Researchers have applied it to the treatment and rehabilitation of disabled children. Literature [4] studied rehabilitation effect of children with cochlear implant treatment based on Gesell scale and analyzed effect of postoperative treatment and rehabilitation systematically and scientifically, providing better guidance for postoperative rehabilitation. In accordance with survey data of the Gesell scale, literature [5] carried out a systematic and comprehensive evaluation on early neurodevelopmental level of children with autism, and the effective treatment plan was designed. Furthermore, literature [6] systematically assessed outcomes and influencing factors of children with three types of developmental disabilities in Beijing according to Gesell scale and implemented targeted rehabilitation treatment and effect tracking for these children, with significant results obtained. For understanding the general situation of mental development of children with suspected mental retardation, a total of 2178 children with suspected mental retardation who completed the Gesell developmental scale were enrolled at West China Second Hospital; language developmental defects are prominent in children with suspected developmental retardation, which are comorbid with different degrees of developmental defects in other functional areas and attention should be paid to the language development of boys. The early intervention of comprehensive mental development based on the language development should be the focus of clinical work right now [7]. Gesell developmental scale can be used as a language development screening tool; it can be used for severity classification and for the children under 2 years old whose language scores of Gesell developmental scale show margin state [8].

This study mainly investigated and analyzed health of 105 disabled children from Disabled Rehabilitation Research Center of minority autonomous region in South China. Subsequently, it systematically evaluated and explored behavioral characteristics of disabled children and various influencing factors for the treatment and rehabilitation. Finally, effective basis and suggestions were proposed for further improving treatment and rehabilitation of disabled children.

## 2. Methodology

### 2.1. Research Objects

This study explored 105 disabled children from Disabled Rehabilitation Research Center of minority autonomous region in the South China, including 84 boys and 21 girls, with an average age of 56.98 months. In addition, there were 48 from Han, 46 from Zhuang, and 11 from other ethnic minorities, so ethnic minorities accounted for 55%. A statistical survey was conducted based on Gesell scale and questionnaires.

### 2.2. Research Process

1. They investigated and collected data from 2018 to 2021, and the data recorded health and development of 105 disabled children. Firstly, questionnaire was imported into an Excel table for preliminary screening and processing, and SPSS22.0 statistical analysis software was used to further analyze data, so as to systematically assess growth and development of disabled children and perform statistical analysis on influencing factors and characteristics.
2. Methodology: the following research methods are introduced to this study: literature review method: based on investigation and analysis of existing research literature, Gesell scale was used as a data collection tool to survey health and development of disabled children in movements [9, 10]. Statistical data analysis: it was adopted to carry out quantitative research and collect data on children's health data released by the Disabled Rehabilitation Research Center of minority autonomous region in South China, in order to initially reveal health and development status of disabled children [10–14].
3. Statistical approach: through input of data and application of SPSS22.0 software, sample variables were explored via descriptive statistical analysis model, mean model, and correlation model provided by SPSS22.0, obtaining analysis statistics and chart to systematically evaluate health and development of disabled children.

### 2.3. Investigation Tools

1. GESSL Health Survey Questionnaire collected movements-related health and development data of disabled children through standard GESSL health questionnaire
2. GESSL Evaluation Form summarized sample information in GESSL health questionnaire with the aid of this tool [15–17]

## 3. Results

### 3.1. Descriptive Statistical Results of Samples

Firstly, in terms of statistics of Gesell scale, SPSS22.0 performed a descriptive statistical analysis of key variable data, with results shown in Table 1.

According to results, standard error of developmental age and developmental quotient variable collected in each ability test interval is within 2.5%, and standard deviation is controlled within 0.2. The distribution of all sample data is in line with general survey results statistics, so it meets research needs.

#### 3.1.1. Statistical Analysis of Comprehensive Disease of Samples

Firstly, results of each ability interval were divided into 6 grades, normal, marginal state, mild developmental retardation, moderate developmental retardation, severe developmental retardation, and very severe developmental retardation, to construct developmental status grade matrix *S* = {0, 1, 2, 3, 4, 5}, where 0 to 5 corresponded to normal development and very severe developmental retardation, respectively.

At the same time, comprehensive disease P was defined as average value of adaptability *p*_*a* *dp*_, big movements *p*_*msup*_, fine movements *p*_*lmps*_, language *p*_*lmps*_, and personal-social *p*_*ps*_. The calculation model is as follows:

(1) $$\begin{array}{c} P=\text{avg}\left\{p_{a\;dp},p_{m\sup},p_{lmps},p_{lan},p_{ps}\right\}. \end{array}$$

Then, based on SPSS software, comprehensive disease was statistically analyzed, and the results are listed in Table 2.

The evaluation of various ability interval indicators meets the expected bootstrap confidence space. The collected Gesell data are highly representative and reliable and can effectively reflect the overall motor development and diseases of disabled children in the study.

According to analysis of comprehensive evaluation data, this study discussed comprehensive ability of samples, finding that comprehensive ability of statistical sample obeyed general normal distribution curve. The ability interval was mainly concentrated in interval of 2.0 to 3.5, that is, areas from mild developmental retardation to moderate developmental retardation, with results shown in Figure 1. The Gesell comprehensive abilities of most disabled children are distributed in this range, and only a few disabled children suffer from severe and very severe diseases.

Through analysis, it was found most of the 105 disabled children suffered from mild and moderate developmental retardation.

From Figure 2, the perspective of age, children aged 3–7 years are affected by more serious comprehensive diseases. Diseases in these age groups are usually serious, especially in moderate and severe patients.

In Figure 3, among analyses of comprehensive diseases, this study described relationship between gender and diseases from the perspective of gender. It shows clearly seen from the cluster diagram that diseases of girls are more serious than that of boys among disabled children. Boys are mainly attacked by moderate developmental retardation, while disabled girls suffer from severe developmental retardation.

### 3.2. Analysis of Performance Characteristics of Diseases

Overall condition had been analyzed from the perspective of comprehensive diseases previously. In order to further explore and study main performance characteristics of sample diseases, this part shall continue to investigate developmental performance in different aspects and discuss correlation.

To begin with, correlation between various factors in ability intervals and the comprehensive diseases was analyzed, in order to explore key performance characteristics of overall condition of disabled children.  Table 3 records correlation test of indicator evaluation of each ability interval and the comprehensive diseases.

According to the above correlation analysis, comprehensive diseases are significantly correlated with five indicators of adaptability, big movements, fine movements, language, and personal-social in the ability test intervals. Fine movements are in particular, whose Pearson correlation value reaches 0.862, and that of other indicators is all above 0.7, showing a significant correlation. Meanwhile, there is also a strong correlation between various indicators in ability test intervals, and the bilateral significance table is above 0.5.

It was necessary to analyze impact and correlation of age and gender on the comprehensive diseases. In Table 4, the results indicated age was significantly correlated with comprehensive diseases, exceeding significance level. But correlation was low between gender and comprehensive diseases, without significant correlation.

## 4. Discussion

According to the above statistical analysis and correlation analysis of sample data, following laws and characteristics are summarized:

1. The overall condition of developmental retardation of disabled children obeys a normal distribution, mainly from mild to moderate developmental retardation, and the developmental retardation is affected by age and gender, to some extent. Among them, children aged 3–7 are easily attacked by moderate and severe developmental retardation. Diseases of girls are more serious than boys, for example, girls usually suffer from severe and very severe developmental retardation. As a whole, a significant correlation is found between age and comprehensive diseases with indicators of ability test intervals. During treatment, rehabilitation should be adopted before the age of 3, in order to control disease deterioration as early as possible [18–20].
2. In terms of correlation, variables of ability test intervals in the Gesell assessment system are significantly correlated with comprehensive disease evaluation variable. There is also a strong correlation among variables of ability test intervals, and comprehensive diseases are obviously affected by adaptability, big movements, fine movements, language, and personal-social. However, according to significance comparison, developmental retardation of overall ability is mainly impacted by fine movements and language that share a significant correlation with age, which is consistent with previous statistical description and analysis. The correlation between diseases and age is unclear, or in other words, boys and girls perform nearly same in specific developmental retardation symptoms. Statistical analysis shows boys generally suffer from moderate and mild developmental retardation, while girls are easily attacked by moderate and severe developmental retardation [21, 22]. In general, language of disabled children in minority areas develops slowly, and they are diagnosed with moderate symptoms. In addition, diseases are significantly correlated with the age. In summary, when formulating treatment and rehabilitation programs, relevant departments should adopt measures according to ages. The focus should be placed on the rehabilitation of fine movements and language. Targeted training and treatment can be provided to disabled children with different degrees of developmental retardation [23].

## 5. Conclusion

This study aims to explore and analyze health development of disabled children in minority areas. Specifically, it focuses on health of disabled children in Guangxi and investigates health status of 105 disabled children from Disabled Rehabilitation Research Center of minority autonomous region in South China [24, 25].

Based on the Gesell scale, it collects health data such as exercise ability and health status of disabled children, analyzes the data in accordance with SPSS software, and constructs comprehensive disease analysis model of disabled children. Moreover, according to five indicator data collected and tested for disabled children (adaptability, big movements, fine movements, language, and personal-social) in Gesell scale, comprehensive disease indicators of the disabled children are calculated and statistically analyzed together with age and gender information. Subsequently, this study analyzed comprehensive diseases and the correlation among various indicators, concluding that most disabled children aged 3–7 are diagnosed with moderate and severe developmental retardation, and retardation level is in obvious normal distribution. At the same time, there is a significant correlation between indicators of ability test interval and measurement indicators with age [26–29].

In view of the above conclusions, this study suggests that targeted treatment and rehabilitation plans should be implemented for disabled children of different ages according to different indicators of ability test interval, which has reference value and significance for improving the treatment level of disabled children and realizing targeted rehabilitation.

## Figures and Tables

**Figure 1:** Distribution curve of comprehensive ability assessment of disabled children sample data.

**Figure 2:** Scatter diagram of distribution of comprehensive disease degree at different ages.

**Figure 3:** Relationship between gender and diseases from the perspective of gender.

**Table 1:** Descriptive statistics of evaluation data of developmental behavior of children aged 0–6.

Ability test interval	Variable	Variable symbol	*N*	Full range	Min	Max	Mean		SD %	Var
			Statistics	Statistics	Statistics	Statistics	Statistics	Standard error %	Statistics	Statistics
——	Age at assessment (months)	V8	105	77.20	19.27	96.47	56.51	1.77	18.26	333.50
Adaptability	Developmental age (months)	V9	105	62.06	6.07	68.13	29.14	1.01	10.39	107.95
	Developmental quotient	V10	105	88.00	15.00	103.00	53.97	1.64	16.78	281.49
Big movements	Developmental age (months)	V12	105	57.63	14.47	72.10	31.83	1.12	11.48	131.89
	Developmental quotient	V13	105	95.00	18.00	113.00	58.77	1.67	17.16	294.56
Fine movements	Developmental age (months)	V15	105	66.27	5.83	72.10	34.04	1.46	14.98	224.43
	Developmental quotient	V16	105	98.00	15.00	113.00	61.55	2.02	20.74	430.25
Language	Developmental age (months)	V18	105	55.54	4.43	59.97	20.32	0.99	10.16	103.31
	Developmental quotient	V19	105	69.00	8.00	77.00	36.64	1.49	15.31	234.29
Personal-social	Developmental age (months)	V21	105	69.07	3.03	72.10	29.00	1.31	13.44	180.75
	Developmental quotient	V22	105	84.00	13.00	97.00	51.34	1.57	16.06	257.92

**Table 2:** Statistical analysis of comprehensive assessment of developmental behaviors of children aged 0–6.

Evaluation item		Statistics	Bootstrap^a^			
			Deviation	SE	95% confidence interval	
					Lower limit	Upper limit
Adaptability	*N*	105	0	0	83	83
	Min	0.00				
	Max	5.00				
	Mean	2.6024	−0.0070	0.1185	2.3614	2.8310
	SD	1.09254	−0.00702	0.08562	0.90838	1.24285
Big movements	*N*	105	0	0	105	105
	Min	0.00				
	Max	5.00				
	Mean	2.3855	−0.0104	0.1146	2.1446	2.5904
	SD	1.05728	−0.00752	0.08294	0.88813	1.21547
Fine movements	*N*	105	0	0	105	105
	Min	0.00				
	Max	5.00				
	Mean	2.2651	−0.0072	0.1425	1.9759	2.5301
	SD	1.28864	−0.00569	0.09202	1.09685	1.46359
Language	*N*	105	0	0	105	105
	Min	1.00				
	Max	5.00				
	Mean	3.6988	−0.0019	0.1125	3.4819	3.9157
	SD	1.05617	−0.00857	0.06152	0.92569	1.16176
Personal-social	*N*	105	0	0	105	105
	Min	0.00				
	Max	5.00				
	Mean	2.7349	−0.0079	0.1052	2.5060	2.9515
	SD	1.00103	−0.00716	0.08424	0.82284	1.15384
Comprehensive disease	*N*	105	0	0	105	105
	Min	0.80				
	Max	5.00				
	Mean	2.7373	−0.0069	0.1002	2.5302	2.9228
	SD	0.92284	−0.00552	0.06257	0.78914	1.03788
Valid *N* (list status)	*N*	105	0	0	105	105

^a^Unless otherwise noted, bootstrap results will be acquired based on 1000 bootstrap samples.

**Table 3:** Correlation analysis of each evaluation indicator of ability interval and comprehensive diseases.

		Adaptability	Big movements	Fine movements	Language	Personal-social	Comprehensive disease
Adaptability	Pearson correlation	1	0.706^*∗∗*^	0.754^*∗∗*^	0.485^*∗∗*^	0.538^*∗∗*^	0.861^*∗∗*^
	Significance (bilateral)		0.000	0.000	0.000	0.000	0.000
	*N*	105	105	105	105	105	105
Big movements	Pearson correlation	0.706^*∗∗*^	1	0.655^*∗∗*^	0.467^*∗∗*^	0.584^*∗∗*^	0.838^*∗∗*^
	Significance (bilateral)	0.000		0.000	0.000	0.000	0.000
	*N*	105	105	105	105	105	105
Fine movements	Pearson correlation	0.754^*∗∗*^	0.655^*∗∗*^	1	0.439^*∗∗*^	0.594^*∗∗*^	0.862^*∗∗*^
	Significance (bilateral)	0.000	0.000		0.000	0.000	0.000
	*N*	105	105	105	105	105	105
Language	Pearson correlation	0.485^*∗∗*^	0.467^*∗∗*^	0.439^*∗∗*^	1	0.544^*∗∗*^	0.711^*∗∗*^
	Significance (bilateral)	0.000	0.000	0.000		0.000	0.000
	*N*	105	105	105	105	105	105
Personal-social	Pearson correlation	0.538^*∗∗*^	0.584^*∗∗*^	0.594^*∗∗*^	0.544^*∗∗*^	1	0.792^*∗∗*^
	Significance (bilateral)	0.000	0.000	0.000	0.000		0.000
	*N*	105	105	105	105	105	105
Comprehensive disease	Pearson correlation	0.861^*∗∗*^	0.838^*∗∗*^	0.862^*∗∗*^	0.711^*∗∗*^	0.792^*∗∗*^	1
	Significance (bilateral)	0.000	0.000	0.000	0.000	0.000	
	*N*	105	105	105	105	105	105

^*∗∗*^Significantly correlated at the 0.01 level (bilateral).

**Table 4:** Correlation analysis of evaluation indicators and comprehensive disease in each ability interval.

		Comprehensive disease	Gender	Age
Comprehensive disease	Pearson correlation	1	−0.153	0.282^*∗∗*^
	Significance (bilateral)		0.119	0.004
	*N*	105	105	105
Gender	Pearson correlation	−0.153	1	0.013
	Significance (bilateral)	0.119		0.892
	*N*	105	105	105
Age	Pearson correlation	0.282^*∗∗*^	0.013	1
	Significance (bilateral)	0.004	0.892	
	*N*	105	105	105

^*∗∗*^Significantly correlated at the 0.01 level (two-sided).

## Data Availability

The datasets used and/or analyzed during the current study are available from the corresponding author on reasonable request.
